The article "The Roles of EXO1 and RPA1 Polymorphisms in Prognosis of Lung Cancer Patients Treated with Platinum-Based Chemotherapy" was published in 2022. Journal: Dis Markers.

# The Roles of EXO1 and RPA1 Polymorphisms in Prognosis of Lung Cancer Patients Treated with Platinum-Based Chemotherapy

**DOI:** 10.1155/2022/3306189

**Published:** 2022-10-13

**Authors:** Jia He, Zhan Wang, Ying Wang, Ting Zou, Xiang-Ping Li, Juan Chen

**Affiliations:** ^1^Department of Pharmacy, Xiangya Hospital, Central South University, Changsha 410008, China; ^2^National Clinical Research Center for Geriatric Disorders, Xiangya Hospital, Central South University, Changsha, Hunan 410008, China; ^3^Department of Medical Oncology, Lung cancer and Gastrointestinal unit, Hunan Cancer Hospital, Affiliated Cancer Hospital of Xiangya School of Medicine, Changsha 410013, China; ^4^Hunan clinical research center in gynecologic cancer, Hunan Cancer Hospital, Affiliated Cancer Hospital of Xiangya School of Medicine, Changsha 410013, China; ^5^National Institution of Drug Clinical Trial, Xiangya Hospital, Central South University, Changsha 410008, China

## Abstract

**Background:**

Lung cancer is one of the major causes of cancer-related mortality worldwide. DNA repair and damage response contribute to genomic instability that accompanies tumor progression. In this study, we focus on evaluating association between DNA repair polymorphisms of EXO1, RPA1, and prognosis in lung cancer patients whom received platinum-based chemotherapy.

**Methods:**

593 lung cancer patients were recruited in this study. We performed genotyping of 19 single nucleotide polymorphisms (SNPs) by Sequenom MassARRAY. Cox regression analysis was used to assess overall survival (OS) and progression-free survival (PFS) among SNP genotypes.

**Results:**

Significant differences in PFS and OS were observed in RPA1 rs5030740, EXO1 rs1776148, and rs1047840. Results showed that patients with CC genotype in rs5030740 (recessive model: *P* = 0.034) had a better PFS. Patients with AA or/and AG genotypes in rs1776148 (additive model: *P* = 0.004; dominant model: *P* = 0.048) and AA genotype in rs1047840 (recessive model: *P* = 0.023) had longer OS. We also demonstrated differences in subgroup analysis between rs5030740, rs1776148, rs1047840, and prognosis.

**Conclusions:**

Our results indicated that EXO1 rs1776148, rs1047840, and RPA1 rs5030740 were significantly associated with prognosis of lung cancer. Rs1776148, rs1047840, and rs5030740 may act as prognosis markers in lung cancer patients with platinum-based chemotherapy.

## 1. Introduction

Lung cancer is one of the most common diseases and one of the leading causes of cancer-related mortality in the world [1]. The statistics estimated that about 1.8 million deaths are due to lung cancer, which accounted for 18.4% of total cancer mortality in 2018 [2]. Despite the advances in diagnosis method that have been used to control the mortality, most patients still have a poor prognosis and high death rates, with an overall 5-year survival rate of 10% to 15% [3]. Currently, it consists of histological subtypes of small lung cancer (SCLC) and non-small lung carcinoma (NSCLC), including adenocarcinoma, squamous cell carcinoma, and large cell lung carcinoma [4, 5]. To date, treatment strategies for lung cancer are surgery, chemotherapy, radiotherapy, target therapies, and immunotherapy [6–8]. And platinum-based chemotherapy still acted as the first-line treatment for lung cancer patients. Besides clinical factors of age, sex, smoking stage, histology, and grade, many genetic polymorphisms also were considered correlation with prognosis in cancer patients. Thus, considering poor prognosis of lung cancer patients, it is crucial to find prognosis markers to develop predictive therapeutic methods.

The article "The Roles of EXO1 and RPA1 Polymorphisms in Prognosis of Lung Cancer Patients Treated with Platinum-Based Chemotherapy" was published in 2022. Journal: Dis Markers.

Previous studies have been identified of the importance of DNA repair and DNA damage response (DDR). The accumulation of mutation in the genome led to genomic instability that accompanies the development of tumors [9, 10]. Genomic alterations in DNA repair genes also play a substantial role in response to chemotherapeutics underlying the genetics of multiple cancers, including breast, colorectal, ovarian, and lung cancer [11–13]. Germline mutations resulted in lung cancer pathogenesis by the constitutive activation of proto-oncogenes, such as the members of the EGFR (ERBB), MYC, and RASfamilies, PIK3CA, NKX2-1, and ALK [11, 14]. Previous study found that single nucleotide polymorphisms (SNPs) in nucleotide excision repair (NER) are associated with progression-free survival, including ERCC1, ERCC6, POLD2, POLE, and XPA [15, 16].

The gene EXO1 (exonuclease 1) was located at the 1q42 to q43 chromosomal region, a RAD2 nuclease family and encoding 846-amino acid protein [17]. It is a multifunctional nuclease and plays crucial roles in DNA mismatch repair (MMR), double-stranded break repair (DSBR), nucleotide excision repair (NER), immunoglobulin maturation, and telomere maintenance [18–21]. Several studies have been conducted on EXO1 related to MMR process by interacting with MSH2 [22]. EXO1 mutations also have been reported concerning different types of tumor and prognosis of cancers, such as breast, ovarian, pancreatic, and lung cancer [23–25]. Luo et al. found that high expression level of the EXO1 is associated with poor OS in breast and prostate cancer patients [26, 27]. It has been studied that high expression of EXO1 could affect OS in colorectal cancer [28]. The canonical RPA heterotrimer (RPA1-3) is an essential coordinator of DNA metabolism that interacts with ssDNA and numerous protein partners to coordinate that has been studied in DNA replication, repair, recombination, and telomere maintenance [29]. RPA1 expression was shown to be increased and correlated with the severity of colon cancer and esophageal carcinoma, suggesting that RPA1 could be used as prognostic indicators or as targets for treatments [30, 31]. In addition, expression of RPA1 has shown markedly correlated with lymphoid tumors and colorectal cancer [32, 33]. PMS1 and PMS2 (the mismatch repair system component) are the fundamental components of mismatch repair (MMR) genes with potential crucial roles in carcinogenesis. The most well-studied variations in certain types of cancers, such as colorectal cancer and breast cancer. However, few studies have been reported on the correlation between PMS and lung cancer.

The article "The Roles of EXO1 and RPA1 Polymorphisms in Prognosis of Lung Cancer Patients Treated with Platinum-Based Chemotherapy" was published in 2022. Journal: Dis Markers.

Currently, genetic polymorphisms in DNA repair are an important factor affecting different cancer, nevertheless association between EXO1, RAP1, PMS1, and PMS2. Therefore, this study is aimed at focusing on the gene polymorphisms of DNA repair pathway genes.

## 2. Method and Materials

### 2.1. Patient Characterization and Data Collection

This study was approved by the Ethics Committee of the Xiangya School of Medicine, Central South University. Patients were recruited from the Affiliated Cancer Hospital or Xiangya Hospital of Central South University (Changsha, Hunan, China) from August 2009 to January 2013. And all patients were provided written informed consent before they participated in this study. To be eligible for the study, patients who had been pathologically diagnosed with lung cancer had to base on the following criteria: (1) the clinical examinations as well as pathological confirmed lung cancer. (2) Lung cancer patients received at least two cycles of platinum-based chemotherapy. (3) Patients without previous surgery, radiotherapy, and target therapies before chemotherapy. Exclusion criteria were pregnancy or lactation, active infection, symptomatic brain or leptomeningeal metastases, and/or previous or concomitant malignancies.

Patients were followed up through outpatients' visits and telephone calls or residence registration. Overall survival (OS) was calculated as the data of diagnosis with lung cancer to the data of death or last follow-up. Progression-free survival (PFS) time was estimated from the pathologically confirmed to the progression of the disease, death without progression, or last clinical follow-up.

### 2.2. SNPs Selection and Genotyping

All of the common genetic variants in EXO1, RPA1, PMS1, and PMS2 involved in DNA damage and repair were selected for genotyping. SNPs must meet the criterion that the minor allele frequency (MAF) ≥ 5% in the HapMap CHB population and call rates >95%. Finally, 19SNPs were genotyped in the patients. The detail information about gene, alleles, call rates, and MAF were listed in Table 1.

The article "The Roles of EXO1 and RPA1 Polymorphisms in Prognosis of Lung Cancer Patients Treated with Platinum-Based Chemotherapy" was published in 2022. Journal: Dis Markers.

The peripheral blood samples (5 mL) were collected from lung cancer patients and stored at -20°C before using. We used FlexiGene DNA Purification Kit to extract the Genomic DNA according to the manufacturer's instructions (Qiagen, Hilden, Germany). The EXO1, RPA1, PMS1, and PMS2 polymorphisms were genotyped by Sequenom MassARRAY system (Sequenom, San Diego, California, USA) through polymerase chain reaction (PCR) system.

### 2.3. Statistical Analysis

The associations of genetic polymorphisms with OS and PFS were evaluated with hazard ratios (HRs) using Cox regression analysis with stepwise selection. The covariates used for adjusted HR for PFS included age, gender, smoking status, histological type, and clinical stage between the OS and PFS. There was no clinical factor significantly related to PFS or OS (Table 2). The log-rank test was used to examine the difference in OS or PFS between groups. Kaplan-Meier plot was used to visualize the results. Three genetic models (Additive model: compares major allele homozygotes versus heterozygotes versus minor allele homozygotes. Dominant model: major allele homozygous verses combined heterozygotes and minor allele homozygous groups. Recessive model: comparing major allele-carrying genotypes with homozygous variant genotype) were constructed, respectively. *P* value <0.05 was considered as statistically significant. All statistical analyses were carried out using the PLINK (version 1.07, http://pngu.mgh.harvard.edu/purcell/plink/) and SPSS 20.0 (SPSS Inc., Chicago, Illinois, USA).

## 3. Results

### 3.1. Clinical Characteristics of Lung Cancer Patients

A total of 593 patients whom received platinum-based chemotherapy were enrolled for this study. The basic descriptive information for lung cancer patients was computed and listed in Table 2. Among them, males were 468 (78.9%) and females were 125 (21.1%). The mean age of patients was 56 years old (range 21 to 77 years). The patients who ever smoke or are current smoker were 366 (61.7%), while never smoker patients were 227 (38.3%). In this study, 122 (20.6%) patients were found in SCLC, 449 (75.7%) patients were NSCLC, and 22 (3.7%) patients were others. There were 68 (11.5%) patients with stage I/II/LD tumors and 519 (87.5%) patients with stages III/IV/ED. The fundamental clinical analysis showed that the median survival time of overall survival (MST-OS) is 4.04 years, and the median survival time of progression-free survival (MST-PFS) is 3.49 years (Table 2). No statistically significant differences were found that PFS/OS of patients and clinical factors.

The article "The Roles of EXO1 and RPA1 Polymorphisms in Prognosis of Lung Cancer Patients Treated with Platinum-Based Chemotherapy" was published in 2022. Journal: Dis Markers.

### 3.2. Association between DNA Repair Genetic Polymorphisms and Prognosis in Lung Cancer Patients

RPA1 rs5030740 genetic polymorphisms were considered to be related to progression-free survival (PFS). For rs5030740 in RPA1, patients who are carrying CC genotype have a better PFS than CT or TT genotype, which median survival time were 3.72, 3.28, and 3.07 years, respectively (recessive model: *P* = 0.034, OR = 0.08, CI = 0.01 − 0.83) (Table 3). Survival analysis was also conducted on log-rank using rs5030740 in RPA1 (Figure 1(a)). In this analysis, the lung cancer patients carrying C allele rs5030740 are regarded as protective alleles in terms of the prolonged PFS.

Two genetic polymorphisms were found to be associated with overall survival (OS), rs1776148 and rs1047840 in EXO1. For rs1776148 in EXO1, patients carrying AA or/and AG genotypes have a prolong OS than GG genotype (additive models: *P* = 0.004, OR = 0.44, 95% CI = 0.25 − 0.77; dominant model: *P* = 0.048, OR = 0.48, 95% CI = 0.23 − 0.99). The median OS duration was 6.96, 4.34, and 4.20 years. For rs1047840 in EXO1, patients carrying AA genotype have a prolong OS than AG and GG genotypes (recessive model: *P* = 0.023, OR = 0.24, 95% CI = 0.07 − 0.82). The median OS duration was 5.43, 4.66, and 3.89 years. In conclusion, lung cancer patients carrying A allele rs1776148 and rs1047840 in EXO1 are regarded as protective alleles in terms of prolonged OS (Figures 1(b)–1(d)). The associations between genetic polymorphisms and PFS/OS are summarized in Table 3.

### 3.3. Stratification Analyses of Association between Polymorphisms and Prognosis in Lung Cancer Patients

Stratification analyses were conducted on association between rs1776148, rs1047840, rs5030740, and prognosis of lung cancer patients. According to clinical characteristics, patients were stratified as age, sex, smoking status, histological type, and stage. Our result found that RPA1 rs5030740 was associated with PFS in patients with age less than 60 years old (additive model: *P* = 0.042, OR = 0.54, 95% CI = 0.30 − 0.98; recessive model: *P* = 0.042, OR = 0.10, 95% CI = 0.01 − 0.92) and patients with clinical stage of III/IV/ED (additive model: *P* = 0.020, OR = 0.90, 95% CI = 0.81 − 0.99; recessive model: *P* = 0.005, OR = 0.57, 95% CI = 0.39 − 0.85) (Figure 2(a)).

For rs1776148 in EXO1, it was correlated with OS in age less than 60 years old in additive model (*P* = 0.027, OR = 0.44, 95% CI = 0.21 − 0.91), male (*P* = 0.003, OR = 0.39, 95% CI = 0.20 − 0.73), never smoked (*P* = 0.044, OR = 0.40, 95% CI = 0.16 − 0.98), ever smoked (*P* = 0.040, OR = 0.46, 95% CI = 0.22 − 0.97), and LUSC patients (*P* = 0.015, OR = 0.39, 95% CI = 0.18 − 0.84). In dominant model, rs1776148 was also related to age under 60 years old (*P* = 0.048, OR = 0.40, 95% CI = 0.16 − 0.99) and LUSC patients (*P* = 0.048, OR = 0.35, 95% CI = 0.12 − 0.99). In recessive model, rs1776148 was related to age more than 60 years old (*P* = 0.005, OR = 0.06, 95% CI = 0.01 − 0.43), male (*P* = 0.001, OR = 0.10, 95% CI = 0.03 − 0.37), never smoked (*P* = 0.034, OR = 0.11, 95% CI = 0.01 − 0.85), smoked (*P* = 0.017, OR = 0.16, 95% CI = 0.03 − 0.72), and LUSC patients (*P* = 0.030, OR = 0.17, 95% CI = 0.03 − 0.85) (Figure 2(b)). EXO1 rs1047840 was associated with OS in recessive model in age less than 60 years old (*P* = 0.006, OR = 0.10, 95% CI = 0.02 − 0.52), male (*P* = 0.016, OR = 0.21, 95% CI = 0.06 − 0.75), and never smoked patients (*P* = 0.034, OR = 0.11, 95% CI = 0.01 − 0.85) (Figure 2(c)).

The article "The Roles of EXO1 and RPA1 Polymorphisms in Prognosis of Lung Cancer Patients Treated with Platinum-Based Chemotherapy" was published in 2022. Journal: Dis Markers.

Furthermore, we also explored the connection between the other 16 SNPs and prognosis in lung cancer patients using subgroups analysis. As shown in Table 4, rs17292622 in RPA1 was associated with PFS in clinical stage in III/IV/ED patients (dominant model: *P* = 0.032, OR = 1.89, 95% CI = 1.06 − 3.38). Rs2228006 in PMS2 was associated with OS in age less than 60 years old in additive genetic model (*P* = 0.027, OR = 0.31, 95% CI = 0.11 − 0.87) and dominant model (*P* = 0.027, OR = 0.31, 95% CI = 0.11 − 0.87). In recessive model, rs1062372 in PMS2 was associated with OS in LUAD patients (*P* = 0.043, OR = 0.16, 95% CI = 0.03 − 0.95) (Table 4).

### 3.4. Base on TCGA Database Examined Prognostic Potential of EXO1 and RPA1 in LUSC and LUAD Cancer

Prognostic analysis is a crucial point of tumor related in recent years. Thus, we further analyzed prognostic significance of EXO1 and RPA1 in diverse tumors compared with normal tissue in Kaplan-Meier plotter database. We focused on detected potential impact of expression of EXO1 and RPA1 on survival rate in LUSC and LUAD via The Cancer Genome Atlas (TCGA) database. Surprisingly, we found that EXO1 expression level had an essential impact on prognosis in LUAD. As shown in Figures 3(a)–3(c), two cohorts of LUAD of lung cancer revealed that higher expression of EXO1 had poorer impact on the PFS and OS (*P* = 0.0033; *P* = 0.0026); however, LUSC had no impact on prognosis (Figures 3(b)–3(d)). Nevertheless, RPA1 expression showed that have little influence on prognosis of LUSC and LUAD. These results suggested that EXO1 might act as an important biomarker that predicts poor prognosis for lung cancer.

The article "The Roles of EXO1 and RPA1 Polymorphisms in Prognosis of Lung Cancer Patients Treated with Platinum-Based Chemotherapy" was published in 2022. Journal: Dis Markers.

## 4. Discussion

In this study, we evaluated whether polymorphisms in DNA damage and repair genes (EXO1, RPA1, PMS1, and PMS2) were associated with prognosis and response to platinum-based chemotherapy in lung cancer patients. Above all, in DNA repair polymorphisms, there was a significant association between EXO1 rs1776148, rs1047840, RPA1 rs5030740, and prognosis in lung cancer. Our results revealed that patients who are carrying rs5030740 C variant allele have a better PFS compared with T allele. Moreover, OS time in lung cancer patients who are carrying rs1776148 A variant allele are longer than patients with G allele. Patients who carry the rs1047840 A variant allele also have a longer OS compared with G allele.

Indeed, DNA replication machinery, exogenous or endogenous mutagen exposures, enzymatic modification of DNA, and defective DNA repair caused genetic alterations [34, 35]. Different mutational and dysfunction processes produce genomic instability, causing tumor progression and metastasis [36, 37]. In the given previous researches, platinum-based drugs could affect tumor sensitivity to platinum drugs by inducing DNA fragmentation and altering DNA repair mechanism. EXO1 activity plays an important role in DNA repair process, cell cycle regulation, and immunoglobulin maturation [38]. The contribution of EXO1 in the maintaining genomic stability during DNA replicative and postreplicative processes is well-established [20, 21]. EXO1 polymorphisms have been reported to be associated with cancer susceptibility. The rs1047840 and rs1776148 have positive association with susceptibility to breast cancer risk [39]. Moreover, large GWAS analysis indicated that specific mutations in EXO1 are more widely occurring in lung cancer, especially in patients with smoking status [40]. Significant differences of allele and genotype distributions were observed in Glu589Lys (rs1047840) of EXO1 between the cases and controls [41]. These previous studies indicated that EXO1 rs1776148 and rs1047840 play an important role in lung cancer and breast cancer. Interestingly, TCGA database indicated that the high expression of EXO1 was significant associated with prognosis in LUAD patients. However, our study results showed that the expression of EXO1 was related to LUSC patients in PFS and OS. The single-stranded DNA binding protein RPA participated in multiple crucial role in DNA repair, DNA metabolism, DNA replication, and DNA resection [33]. Moreover, RPA depletion eliminated EXO1-dependent extensive resection pathways and synergized with mre11 to prevent end resection [42]. DNA resection by EXO1 is probably inhibited by the DNA binders RPA, Ku70/80, and/or C-terminal-binding protein interacting protein (CtIP) [20, 43, 44]. Overexpression RPA1 was related to poor clinical outcomes in bladder cancer and esophageal cancer [30, 45]. Rs5030740 was located in the 3′-UTR of RPA1, which is carrying C allele markedly associated with poor DCR and prognosis compared to those with the T allele in colorectal cancer [29].

The article "The Roles of EXO1 and RPA1 Polymorphisms in Prognosis of Lung Cancer Patients Treated with Platinum-Based Chemotherapy" was published in 2022. Journal: Dis Markers.

Here, our results also revealed that AA genotype of rs1776148 with platinum-based chemotherapy had better clinical prognosis compared with those of AG and GG genotypes. Further studies indicated younger age (≤60), male, never smoked or smoked, and LUSC patients are related to OS time. Rs1047840 is located on exon12 and its change causes the 589th amino acid of the EXO1 protein product to be altered from lysine to glutamic acid [40]. We also found that rs1047840 was associated with OS. For rs1047840, we further analyzed the stratified analysis, age less than 60 years old, male, and never smoked patients, were associated with prognosis.

Our results indicated that CC genotype of rs5030740 with platinum-based chemotherapy had better clinical outcomes compared with those of CT and TT genotypes. In detail, rs5030740 polymorphisms in the subgroups of age less than 60 and clinical stages in III/IV/ED patients are associated with prognosis in the stratified analysis. Expect for the polymorphisms of EXO1 rs1776148, rs1047840, and RPA1 rs5030740, we also found other polymorphisms were associated with prognosis in some subgroups, such as RPA1rs17292622, was related to PFS in patients who are in the clinical stages of III/IV/ED. PMS2 rs2228006 was associated with OS time in younger patient who is less than 60 years old, and rs1062372 was associated with OS time in LUAD patients.

However, this study still have several limitations. First, further large-scale independent studies are required to validate our results. Second, statistical significance was not maintained when multiple testing correction was conducted. Third, expression studies of genetic polymorphisms identified need to further study, which would be helpful to demonstrate the results of this study.

In conclusion, we identified several genetic polymorphisms associated with prognosis in lung cancer patients who received platinum-based chemotherapy. The genetic polymorphisms of rs5030740 C variant allele had a better PFS compared with T allele. The genetic polymorphisms of rs1776148 and rs1047840 A variant allele are longer than patients with G allele. The genotypes of RPA1 rs5030740, EXO1 rs1776148, and rs1047840 may be a biomarker contribute to predict the prognosis of platinum-based chemotherapy lung cancer patients.

## Figures and Tables

**Figure 1:** The RPA1 rs5030740, EXO1 rs1776148, and rs1047840 polymorphisms are significantly associated with prognosis of lung cancer treated with platinum-based chemotherapy. (a) The RPA1 rs5030740 is significantly associated with PFS in lung cancer patients treated with platinum-based chemotherapy in recessive model. (b) The EXO1 rs1776148 is significantly associated with OS in lung cancer patients treated with platinum-based chemotherapy in additive model. (c) The EXO1 rs1776148 is significantly associated with OS in lung cancer patients treated with platinum-based chemotherapy in dominant model. (d) The EXO1 rs1047840 is significantly associated with OS in lung cancer patients treated with platinum-based chemotherapy in recessive model.

The article "The Roles of EXO1 and RPA1 Polymorphisms in Prognosis of Lung Cancer Patients Treated with Platinum-Based Chemotherapy" was published in 2022. Journal: Dis Markers.

**Figure 2:** Stratification analyses of the associations of DNA repair polymorphisms with prognosis in lung cancer patients. (a) RPA1 rs5030740 polymorphisms is significantly associated with the PFS; (b) EXO1 rs1776148 polymorphisms is significantly associated with the OS; (c) EXO1 rs1047840 polymorphisms is significantly associated with OS.

**Figure 3:** Association between EXO1 expression and prognosis in LUSC and LUAD in TCGA database. (a) LUSC of lung cancer in different expression of EXO1 had no significant impact on the PFS; (b) LUAD of lung cancer in different expression of EXO1 had essential impact on the PFS; (c) LUSC of lung cancer in different expression of EXO1 had no significant impact on the OS; (d) LUAD of lung cancer in different expression of EXO1 had essential impact on the OS.

**Table 1:** The 19 single nucleotide polymorphisms examined in this study.

Gene	SNPs	Alleles	MAF	Call rates (%)
EXO1	rs1047840	G/AC	0.35	97.03
EXO1	rs1776148	A/GT	0.32	97.78
EXO1	rs735943	A/G	0.36	97.78
PMS1	rs5742933	G/AC	0.22	96.30
PMS2	rs1062372	C/AGT	0.23	95.56
PMS2	rs2228006	T/ACG	0.12	99.01
RPA1	rs17292622	G/AT	0.22	98.84
RPA1	rs17339382	G/A	0.09	92.28
RPA1	rs3744768	G/A	0.20	98.55
RPA1	rs12727	G/C	0.24	98.26
RPA1	rs17339395	G/ACT	0.22	98.55
RPA1	rs9914073	A/CG	0.23	98.26
RPA1	rs9082	T/C	0.23	98.84
RPA1	rs3744766	C/G	0.22	98.84
RPA1	rs1131636	C/AGT	0.46	98.84
RPA1	rs5030740	C/AGT	0.30	99.42
RPA1	rs3744767	T/C	0.24	99.42
RPA1	rs3744769	C/AGT	0.22	97.69
RPA1	rs17734	C/T	0.43	99.42

MAF: minor allele frequency.

**Table 2:** Main clinical characteristics of lung cancer patients and prognosis analysis.

Characteristics	Patients *N* (%)	Death *N* (%)	MST-OS (year)	P	MST-PFS (year)	*P*
Total	593	416	4.04		3.49	
Age (years)						
≤60	412 (69.4)	280 (67.3)	4.38	0.822	3.43	0.692
>60	181 (30.5)	136 (32.6)	4.65		3.75	
Sex						
Male	468 (78.9)	335 (80.5)	4.38	0.082	3.45	0.449
Female	125 (21.1)	80 (19.2)	4.53		3.43	
Smoking status						
Nonsmoker	227 (38.3)	149 (35.8)	4.53	0.132	3.28	0.411
Smoker	366 (61.7)	265 (63.7)	4.36		3.45	
Histology						
NSCLC	449 (75.7)	359 (76.4)	4.68	0.361	4.44	0.093
SCLC	122 (20.6)	93 (8.3)	4.42		4.01	
Others	22 (3.7)	18 (3.8)	3.81		4.10	
Stage						
I/II/LD	68 (11.5)	44 (10.6)	4.62	0.345	4.30	0.558
III/IV/ED	519 (87.5)	363 (87.3)	4.31		3.41	

NSCLC: non-small-cell lung cancer; SCLC: small cell lung cancer; LUSC: squamous cell carcinoma; LUAD: adenocarcinoma.

The article "The Roles of EXO1 and RPA1 Polymorphisms in Prognosis of Lung Cancer Patients Treated with Platinum-Based Chemotherapy" was published in 2022. Journal: Dis Markers.

**Table 3:** Association between DNA repair polymorphisms and platinum-based chemotherapy prognosis.

PFS/OS	Gene	Polymorphism	Genotype	MST (year)	Additive		Dominant		Recessive	
					OR (95% CI)	*P*	OR (95% CI)	*P*	OR (95% CI)	*P*
PFS	RPA1	rs5030740	CC	3.72	0.67 (0.40-1.13)	0.136	0.76 (0.43-1.34)	0.341	0.08 (0.01-0.83)	**0.034**
			CT	3.28						
			TT	3.07						
OS	EXO1	rs1776148	AA	6.96	0.44 (0.25-0.77)	**0.004**	0.48 (0.23-0.99)	**0.048**		
			AG	4.34						
			GG	4.20						
	EXO1	rs1047840	AA	5.43	0.67 (0.37-1.20)	0.177	0.80 (0.39-1.66)	0.551	0.24 (0.07-0.82)	**0.023**
			AG	4.66						
			GG	3.89						

MST: median survival time. Additive model: comparison between minor allele subjects and major allele subjects. Dominant model: comparison between minor allele carriers and major homozygous subjects. Recessive model: comparison between major allele carriers and minor homozygous subjects. ^∗^**P** < 0.05.

**Table 4:** Stratification analyses of association between polymorphisms and PFS or OS in lung cancer patients.

PFS/OS	Polymorphism	Genotype	Subgroup	Additive		Dominant		Recessive	
				OR (95% CI)	*P*	OR (95% CI)	*P*	OR (95% CI)	*P*
PFS	rs17292622	RPA1	TNM2	1.56 (0.98-2.48)	0.060	1.89 (1.06-3.38)	**0.032**	1.34 (0.49-3.67)	0.563
OS	rs2228006	PMS2	≤60	0.31 (0.11-0.87)	**0.027**	0.31 (0.11-0.87)	**0.027**		
	rs1062372	PMS2	LUAD	0.49 (0.20-1.20)	0.121	0.58 (0.18-1.81)	0.347	0.16 (0.03-0.95)	**0.043**

Additive model: comparison between minor allele subjects and major allele subjects. Dominant model: comparison between minor allele carriers and major homozygous subjects. Recessive model: comparison between major allele carriers and minor homozygous subjects. OR: odds ratio; CI: confidence interval. ^∗^**P** < 0.05.

## Data Availability

The data will be made available on reasonable request.
